The article "Correlations between Clinical Characteristics and Prognosis in Patients with Grade II Glioma" was retracted in 2023. Reasons: unreliable results or conclusions; lack of ethics approval or compliance; concerns about the data; concerns about the peer review.

# Correlations between Clinical Characteristics and Prognosis in Patients with Grade II Glioma

**DOI:** 10.1155/2021/5873213

**Published:** 2021-10-13

**Authors:** Liang Ning, Weidong Liang, Hongjun Guo, Jun Liu, Lanjun Xie

**Affiliations:** Fuyang People's Hospital, Fuyang, China

## Abstract

**Objective:**

Grade II gliomas are mostly astrocytomas and oligodendrocytomas. The treatment method is mainly surgery, combined with chemotherapy and radiotherapy. According to statistics, young patients under the age of 40 years with grade II gliomas have a 50% chance of more than 5-year survival through reasonable treatment and normal eating habits. The survival time of middle-aged and elderly patients over 40 years old is about 2-3 years under the same conditions. The study aimed at analyzing the clinical characteristics and prognostic factors of 60 patients with glioma.

**Methods:**

A total of 60 patients diagnosed pathologically with grade II glioma according to the World Health Organization (WHO) classification in 2007 admitted into our hospital from January 2016 to December 2016 were retrospectively analyzed. The Kaplan–Meier curve was plotted to reflect 5-year survival according to patients' clinical characteristics. The Cox regression model was used to analyze prognostic factors of grade II glioma.

**Results:**

Preoperative KPS scores <60, 60–80, and >80 accounted for 25.00% (15/60), 40.00% (24/60), and 35.00% (21/60), respectively. The largest tumor diameter LTD was less than 5 cm revealed in 60.00% patients, of which astrocytoma accounted for 65.00%. Subventricular zone (SVZ) expansion occurred in 23.33% of the patients and peritumoral edema occurred in 16.67% of the patients. The median follow-up time was 54 months. 5-year overall survival and progression-free survival rates of all patients were 70.0% and 56.7%, respectively. The Cox regression model indicated SVZ expansion, surgical resections, and recurrence were the independent prognostic factors of grade II glioma.

**Conclusion:**

These data suggested that SVZ expansion, surgical resections, and recurrence were independent factors affecting the prognosis of grade II glioma. According to the above clinical indexes of patients, individualized therapies can be established to prolong the survival time of patients.

## 1. Introduction

Glioma refers to the most common primary malignant brain tumor, which can occur anywhere in the central nervous system, but mainly in the brain and glial tissue [1]. The incidence rate of glioma is increasing in younger adults, and it possesses the characteristics of normal neuroglia cell and is usually named according to these similarities. According to World Health Organization (WHO) classification in 2007 [2], the main glioma groups are represented by astrocytoma, oligodendroglioma, and a mix of these 2 cell types, ependymal tumors, and neuronal and mixed neuronal-glial tumors. The glioma can be classified as grades I–IV based on the malignant behavior. It includes more limited grade I tumor, such as pilocytic astrocytoma, pleomorphic xanthoastrocytoma, and subependymal giant cell astrocytoma. The most common histological types of adult gliomas include grade II astrocytoma and oligodendroglioma, grade III anaplastic oligodendroglioma, anaplastic astrocytoma, anaplastic ependymoma, and grade IV glioblastoma. However, there is no consistent definition of glioma as a larger histological category [3, 4]. Glioma accounts for around 81% of malignant brain tumors, of which about 3 cases out of 100,000 people suffer from glioblastoma (grade IV) each year [5]. The median survival of glioblastoma is less than 2 years after surgery resection combined with chemoradiotherapy [6]. Certain glioma subtypes cause significant mortality rate, which is disproportionate to incidence rate.

The article "Correlations between Clinical Characteristics and Prognosis in Patients with Grade II Glioma" was retracted in 2023. Reasons: unreliable results or conclusions; lack of ethics approval or compliance; concerns about the data; concerns about the peer review.

At present, many potential factors, such as genetic factors [7] and ionizing radiation exposures [8], have been proved to be related to the increased risk of glioma occurrence [9]. In general, surgical resection is the main treatment for glioma, which reduces intracranial pressure, attenuates neurological symptoms, and prolongs survival time of patients. Low-grade glioma (grades II and III) are considered as slow-processing brain tumor, many of which eventually turn into more aggressive tumor. Patients with low-grade glioma showed better prognosis and indicated certain sensitivity to treatment, which depends on molecular subtypes [10]. The applications of chemotherapy, radiotherapy, and chemoradiotherapy depend on clinical and molecular risk factors after surgery resection in low-grade glioma patients [11, 12]. Although it has been proven that, compared with high-grade gliomas patients, the low-grade glioma patients have relative long survival time which might be more than 15 years [13], the best treatment for low-grade glioma patients is controversial since the differences of the prognostic outcomes are reported by previous studies. In view of this, this study retrospectively analyzed the clinical data of 63 patients with grade II glioma in our hospital and focused on the risk factors affecting their prognosis, so as to provide reference for the clinical treatment of grade II glioma.

## 2. Methods

### 2.1. Study Subjects

The study was performed on the patients with grade II gliomas diagnosed by histopathology and immunohistochemistry and receiving surgical resections in our hospital from January 2016 to December 2016. The study subjects were included if they were eligible for the following inclusion criteria: grade II gliomas according to the 2007 Revised WHO Classification of Tumors of the Central Nervous System, complete clinical data and imaging data, successful follow-up, and signed the informed content. The patients with other malignancies, severe coronary heart disease, congenital heart disease, diabetes and hypertension, and receiving previous chemoradiotherapy regimes and antitumor therapy were excluded. The study was approved by the Ethics Committee of Fuyang People's Hospital. Each subject signed the informed content.

The article "Correlations between Clinical Characteristics and Prognosis in Patients with Grade II Glioma" was retracted in 2023. Reasons: unreliable results or conclusions; lack of ethics approval or compliance; concerns about the data; concerns about the peer review.

### 2.2. Data Collection

According to clinical medical records and follow-up data, the following information of each patient was recorded: (a) clinical characteristics including gender, age, preoperative Karnofsky performance scale (KPS) score, largest tumor diameter (LTD) by CT or MRI before operation (in case of multiple lesions, it was calculated by the sum of the maximum single diameter of each lesion), peritumoral edema, pathological type, and lesion conditions such as multiple lesion, location of largest lesion, and subventricular zone (SVZ) expansion; (b) treatment information including surgical resections, radiotherapy, and chemotherapy; and (c) patient survival including overall survival, progression-free survival, and time of tumor recurrence.

### 2.3. Postoperative Chemoradiotherapy Regimes

In this study, 3-dimensional conformal radiotherapy was carried out 2–4 weeks after surgery when surgical wounds were closured. Before radiotherapy, all patients were fixed on a computer tomography (CT) simulator with a plastic head mold. The scanning was performed by an enhanced CT with a layer thickness of 3 mm, and the scanned image was transmitted to the three-dimensional treatment planning system (3D-TPS). The postoperative residual lesions and surgical cavity, shown in T2-weighted image (T2WI) by magnetic resonance imaging (MRI), were considered as gross tumor volume (GTV). 1-2 cm outside the edge of clinical target volume (CTV) was defined as planning target volume (PTV). The target area covered 90% isodose curve, which was taken as the reference dose curve. Fractionated radiation dose was 2 Gy/time. Radiation area was confirmed when the dose reached 50 Gy. With 0.8–1.0 cm outside the edge of CTV and 50–66 Gy dose in total, radiotherapy was started with 6-MV X-ray given by the Varian linear accelerator (Varian Medical Systems, Palo Alto, CA, USA). In the presence of intracranial hypertension symptoms, such as headache, dizziness, and vomiting; during the therapy, antihypertensive therapy should be carried out. In general, 20% mannitol injection, glycerol fructose or glycerol saline mixture, and the dose and frequency of use were selected according to the severity of symptoms. At the same time, blood pressure or blood sugar should be observed in patients with diabetes or hypertension receiving dexamethasone and mannitol. For the sake of prevention of electrolyte imbalance, potassium concentration in serum was observed if the patients received dehydrating agent. Generally, the symptoms of patients can be significantly relieved after intracranial pressure was reduced. Chemotherapy was performed 2–4 weeks after surgery, 4–6 cycles in total, with 28 d for each cycle. The patients required receiving chemotherapy, or their families were informed of potential toxic and side effects caused by chemical drugs. The daily oral dose of temozolomide was 50–75 mg/m^2^. Generally, temozolomide has no obvious toxic and side effects, such as bone marrow suppression and gastrointestinal reactions on patients, and mild side effects could be tolerated or relieved by corresponding treatments. The withdrawal of temozolomide was confirmed when the patients failed to tolerate severe adverse reactions or the patient's condition progresses during the medication.

The article "Correlations between Clinical Characteristics and Prognosis in Patients with Grade II Glioma" was retracted in 2023. Reasons: unreliable results or conclusions; lack of ethics approval or compliance; concerns about the data; concerns about the peer review.

### 2.4. Follow-Up

The patients returned to the hospital for reexamination every 3 months until 2 years after the end of treatment and then received reexamination every 6 months. Reexamination basically included physical examination, brain CT or MRI, and other examinations according to their own symptoms. Progression-free survival (PFS) refers to the time from the date of surgical treatment to the discovery of disease progression or the latest follow-up. Overall survival (OS) refers to the time from the date of surgical treatment to the patient's death or the latest follow-up.

### 2.5. Statistical Analysis

SPSS 19.0 software was used for statistical analysis with test level *α* = 0.05. The counting data were described by *N* or %. The Kaplan–Meier method was applied to analyze the prognosis of patient survival. The log-rank test was carried out to compare the survival rate. The Cox regression model was used for the analysis of prognostic factors. Variance inflation factor (VIF) was applied to reflect colinearity. *P* < 0.05 indicated the difference was statistically significant.

## 3. Results

### 3.1. Baseline Characteristics of Eligible Patients with Grade II Glioma

A total of 60 patients with grade II glioma were included in this study, with 33 cases of man and 27 cases of woman, ranging from 17 to 69 years old, of which patients under 40 years of age and over 40 years of age were both 30 cases (50%). The patients with preoperative KPS scores <60, 60–80, and >80 accounted for 25.00% (15/60), 40.00% (24/60), and 35.00% (21/60), respectively. The LTD not less than 5 cm was found in 24 cases of patients and less than 5 cm in 36 cases of patients. The patients with pathological types of astrocytoma and oligodendroglioma alone or both accounted for 65.00% (39/60), 21.67% (13/60), and 13.33% (8/60), respectively. The cases of patients with SVZ expansion and peritumoral edema were 14 (14/16, 23.33%) and 10 (10/60, 16.67%), respectively. The largest lesion located in the temporal lobe, frontal lobe, parietal lobe, occipital lobe, corpus callosum, thalamus, pons, cerebellum, and insula occupied 25.00% (15/60), 50.00% (30/60), 11.67% (7/60), 3.33% (2/60), 3.33% (2/60), 1.67% (1/60), 1.67% (1/60), 1.67% (1/60), and 1.67% (1/60), respectively.

The article "Correlations between Clinical Characteristics and Prognosis in Patients with Grade II Glioma" was retracted in 2023. Reasons: unreliable results or conclusions; lack of ethics approval or compliance; concerns about the data; concerns about the peer review.

### 3.2. Classification of Patients with Grade II Glioma according to Surgical Resections and following Chemoradiotherapy

All patients underwent surgical resection. Among them, 37 patients (61.67%) were given total resection and 23 patients (38.33%) were given partial resection. After surgery, 48 patients (80%) received radiotherapy, of which 28 cases (58.33%) had less than 30 days of duration between surgery to radiotherapy and 20 cases (41.67%) had more than 30 days of duration. More than 54 Gy irradiation dosages were found in 25 patients (52.08%). There were 14 patients (23.33%) receiving postoperative temozolomide-based chemoradiotherapy.

### 3.3. Survival Analysis of the Patients with Grade II Glioma

Among 60 patients, there were 18 cases of death and 26 cases of recurrence based on 54 months of median follow-up. After analysis by the Kaplan–Meier method, the 5-year OS was 70.0% and the 5-year PFS rate was 56.7%, as shown in Figure 1.

### 3.4. Univariate Analysis of Clinical Characteristics Affecting the Prognosis of Patients with Grade II Glioma

As given in Table 1, it was observed that the 5-year overall survival of 60 patients was significantly different based on clinical characteristics, such as gender, age, pathological type, peritumoral edema, SVZ expansion, peritumoral edema surgical resections, and recurrence (*P* < 0.05). Results showed that female patients, the patients aged less than 40 years, the patients receiving total resection, and the patients without tumor recurrence exhibited significantly higher 5-year overall survival rates than male patients, the patients aged more than 40 years, the patients receiving partial resection, and the patients with tumor recurrence (*P* < 0.05). The patients with oligodendroglioma or mixed oligodendroglioma showed remarkably higher 5-year overall survival rates than those with astrocytoma (*P* < 0.05). However, slight difference was found between the patients with oligodendroglioma and mixed oligodendroglioma (*P* > 0.05). The patients with SVZ expansion and peritumoral edema showed remarkable lower survival rates than those without (*P* < 0.05).

The article "Correlations between Clinical Characteristics and Prognosis in Patients with Grade II Glioma" was retracted in 2023. Reasons: unreliable results or conclusions; lack of ethics approval or compliance; concerns about the data; concerns about the peer review.

### 3.5. Independent Risk Factors Affecting the Prognosis of the Patients with Grade II Glioma

The Cox regression model analysis was performed with survival time as time and death as status, gender (female = 1; male = 2), age (<40 years = 1; ≥40 years = 2), pathological type (nonastrocytoma = 0; astrocytoma = 1), SVZ expansion (no = 0; yes = 1), peritumoral edema (yes = 1; no = 0), surgical resections (total resection = 0; partial resection = 1), and recurrence (yes = 1; no = 0). The Cox regression model observed that SVZ expansion, surgical resections, and recurrence were the independent risk factors affecting the prognosis of the patients with grade II glioma (*P* < 0.05, Table 2, Figures 2–4), and each VIF was less than 3.

## 4. Discussion

Glioma is a malignant tumor disease originated from brain glial cells. As a common intracranial primary tumor disease, it accounts for about 31% of all intracranial tumors and 81% of malignant intracranial tumors [1]. Glioma is classified into four grades involving grades I, II, III, and IV reported by the WHO. Low-grade glioma includes grades I and II. Grades III and IV belong to high-grade glioma, which are more malignant than grades I and II. In addition, the most common subtypes of glioma involve astrocytoma (grades I–IV), oligodendroglioma (grades II-III), oligoastrocytoma (grades II-III), and glioblastoma (grade IV) [3]. Surgical resection acts a central role in treatment of glioma. Although glioma is a typical malignant tumor, not all types of tumors are malignant. Previous studies have found that the patients with low-grade glioma have long survival time after surgical care [14, 15].

Tons of reports have been done on the factors affecting the prognosis of patients with gliomas, but with relative few reports on the factors affecting the prognosis of grade II gliomas. Furthermore, the conclusions of prognostic factors obtained from reports are varied due to the differences of research objects, sample size, variable collection, and other factors [16, 17]. In order to further supplement and improve the clinical treatment of grade II glioma, the clinical characteristics and prognostic factors of 60 patients with grade II gliomas were analyzed to find their correlations in this study.

The Kaplan–Meier method indicated that the 5-year overall survival was 70.0% and the 5-year progression-free survival was 56.7%. Another study on child low-grade glioma also revealed that the 5-year overall survival and progression-free survival were 90.6 ± 4.7% and 54.3 ± 8.4%, respectively [18]. These findings proved that low-grade glioma patients who underwent treatment run lower risk of death. The prognosis analysis showed that overall survival was associated with various factors, including gender, age, tumor recurrence, tumor type, peritumoral edema, and SVZ invasion. The Cox regression model also showed that SVZ expansion, surgical resections, and tumor recurrence were independent risk factors affecting prognosis outcomes. Surgical resection plays a central role in the treatment of glioma, which can delay tumor malignant transformation and recurrence [19]. In this study, the overall survival of patients with total resection was significantly higher than that of patients with partial resection. The findings were similar to previous study, indicating the patients with low-grade glioma who underwent partial resection run higher risk of tumor recurrence and death compared to the patients received total resection [20]. Total resection for grade II glioma associated with higher overall survival might due to minor tumor residue, which can effectively inhibit the proliferation of subclinical lesions through radiotherapy or chemotherapy [21]. SVZ is distributed in the lateral wall of lateral ventricle within 3–5 mm, which is considered as neural stem cell niche. SVZ is considered to be a tumor reservoir for a series of high-grade gliomas including adult glioblastoma [22]. SVZ involvement in the context of gliomas has been confirmed to be related to a shorter patient survival [23, 24] and a higher risk of tumor recurrence [25, 26]. The present study also demonstrated that the overall survival of patients with grade II gliomas with SVZ expansion was significantly higher than that of patients without SVZ expansion. The reason is that when the tumor tissue involves SVZ, abnormal neural stem cell formation occurs in the lower region of SVZ, which can not only change the biological malignant behavior of the tumor but also promote tumor proliferation and invasion through the regulation of the CXCL12 signaling pathway [27].

The article "Correlations between Clinical Characteristics and Prognosis in Patients with Grade II Glioma" was retracted in 2023. Reasons: unreliable results or conclusions; lack of ethics approval or compliance; concerns about the data; concerns about the peer review.

In summary, astrocytoma is the most common grade II glioma, and the largest lesions are mostly distributed in the frontal lobe. SVZ invasion, surgical resections, and postoperative recurrence are the independent factors affecting the survival of grade II glioma. However, some limitations such as small sample size which might lower the reliability of experimental data exist in the study. Further studies involving large sample capacity and intensive interventions should be done in near future. Anyway, total resection should be carried out for grade II glioma patients as far as possible to reduce residual tumor cells and strengthen regular follow-up after operation to find recurrent lesions in time and actively intervene.

## Figures and Tables

**Figure 1:** Kaplan–Meier curves showing the survival of 60 patients with grade II gliomas. (a) Overall survival analysis. (b) Progression-free survival analysis.

**Figure 2:** The Kaplan–Meier curves showing the survival of 60 patients with grade II gliomas based on the presence of SVZ expansion.

**Figure 3:** The Kaplan–Meier curves showing the survival of 60 patients with grade II gliomas based on total or partial resection surgery.

**Figure 4:** The Kaplan–Meier curves showing the survival of 60 patients with grade II gliomas based on the occurrence of tumor recurrence.

**Table 1:** Univariate analysis of prognosis of the patients with grade II glioma.

Factors		Cases	5-Year overall survival (%)	*X* ^2^	*P*
Gender	Male	33	57.6	5.018	0.025
	Female	27	85.0		

Age	<40	30	90.0	10.844	0.001
	≥40	30	50.0		

Preoperative KPS scores	<60	15	80.0	3.143	0.208
	60–80	24	75.0		
	>80	21	57.1		

LTD	≥5 cm	24	75.0	0.505	0.477
	<5 cm	36	66.7		

Pathological type	Astrocytoma	39	59.0	6.586	0.037
	Oligodendroglioma	13	84.6		
	Mixed of these two types	8	100.00		

SVZ expansion	Yes	14	95.0	84.106	≤0.001
	No	46	0.00		

Peritumoral edema	Yes	10	84.0	37.069	≤0.001
	No	50	0.00		

Multiple lesions	Yes	58	100.00	0.737	0.391
	No	2	69.0		

Surgical resections	Total resection	37	86.5	13.455	≤0.001
	Partial resection	23	43.5		

Residual tumor volume	≥3 mL	20	75.0	0.206	0.650
	<3 mL	40	67.5		

Radiotherapy	Yes	48	68.7	0.213	0.644
	No	12	75.0		

Duration between surgery to radiotherapy	>30 d	28	75.0	0.263	0.608
	≤30 d	20	65.6		

Irradiation dosage	45–54 Gy	23	78.3	1.936	0.164
	>54 Gy	25	60.0		

Chemotherapy	Yes	14	64.3	1.182	0.670
	No	46	71.7		

Tumor recurrence	Yes	26	42.3	18.037	≤0.001
	No	34	91.2		

KPS, Karnofsky performance scale; SVZ, subventricular zone.

**Table 2:** Cox regression model of prognosis in the patients with grade II glioma.

Variable	*B*	SE	Wald	*P*	Exp (*B*)	95.0% CI applied to Exp (*B*)		VIF
						Lower limits	Upper limits	
Gender	1.703	1.021	2.782	0.096	5.490	0.742	40.616	2.002
Age	1.317	0.948	1.930	0.165	3.732	0.582	23.929	1.677
Astrocytoma	1.327	1.003	1.830	0.176	3.885	0.544	27.710	2.473
SVZ expansion	1.024	0.327	9.806	0.001	2.784	1.467	5.285	1.511
Peritumoral edema	0.277	0.729	0.097	0.755	1.255	0.301	5.237	1.887
Surgical resections	1.669	0.667	6.261	0.012	5.307	1.436	19.615	1.790
Tumor recurrence	1.024	0.336	9.288	0.002	2.784	1.441	5.379	0.715

SVZ, subventricular zone; *B*, regression coefficient; SE, standard error; Wald, statistics; Exp (*B*), risk coefficient; 95.0% CI, 95.0% confidence interval; VIF, variance inflation factor.

The article "Correlations between Clinical Characteristics and Prognosis in Patients with Grade II Glioma" was retracted in 2023. Reasons: unreliable results or conclusions; lack of ethics approval or compliance; concerns about the data; concerns about the peer review.

## Data Availability

The data used to support the findings of this study are included within the article.
